This article has been retracted.

# Application Value of a Deep Convolutional Neural Network Model for Cytological Assessment of Thyroid Nodules

**DOI:** 10.1155/2021/6076135

**Published:** 2021-11-09

**Authors:** Ying Ren, Yu He, Linghua Cong

**Affiliations:** Department of Pathology, The Affiliated People's Hospital of Ningbo University, Ningbo 315000, Zhejiang Province, China

## Abstract

**Objective:**

To investigate the application value of a deep convolutional neural network (CNN) model for cytological assessment of thyroid nodules.

**Methods:**

117 patients with thyroid nodules who underwent thyroid cytology examination in the Affiliated People's Hospital of Ningbo University between January 2017 and December 2019 were included in this study. 100 papillary thyroid cancer samples and 100 nonmalignant samples were collected respectively. The sample images were translated vertically and horizontally. Thus, 900 images were separately created in the vertical and horizontal directions. The sample images were randomly divided into training samples (*n* = 1260) and test samples (*n* = 540) at the ratio of 7 : 3 per the training sample to test sample. According to the training samples, the pretrained deep convolutional neural network architecture Resnet50 was trained and fine-tuned. A convolutional neural network-based computer-aided detection (CNN-CAD) system was constructed to perform full-length scan of the test sample slices. The ability of CNN-CAD to screen malignant tumors was analyzed using the threshold setting method. Eighty pathological images were collected from patients who received treatment between January 2020 and May 2020 and used to verify the value of CNN in the screening of malignant thyroid nodules as verification set.

**Results:**

With the number of iterations increasing, the training and verification loss of CNN model gradually decreased and tended to be stable, and the training and verification accuracy of CNN model gradually increased and tended to be stable. The average loss rate of training samples determined by the CNN model was (22.35 ± 0.62) %, and the average loss rate of test samples determined by the CNN model was (26.41 ± 3.37) %. The average accuracy rate of training samples determined by the CNN model was (91.04 ± 2.11) %, and the average accuracy rate of test samples determined by the CNN model was (91.26 ± 1.02)%.

**Conclusion:**

A CNN model exhibits a high value in the cytological diagnosis of thyroid diseases which can be used for the cytological diagnosis of malignant thyroid tumor in the clinic.

## 1. Introduction

Thyroid nodules are common clinical diseases which can be toughed in about 5% of women and about 1% of men. The incidence rate of nonpalpable thyroid nodules detected by ultrasound is 20%–76% [1,2]. Malignant thyroid nodules are one of the top 10 malignant tumors and account for 1.1% of all malignant tumors [3]. Ultrasound-guided fine-needle aspiration cytology (US-FNAC) can be used for differential diagnosis of malignant thyroid nodules [2]. Diagnosis of thyroid nodules by US-FNAC depends on doctor's experience. The uncertainty of the diagnosis after US-FNAC is likely attributable to doctor's insufficient experience. Improving the diagnostic accuracy of US-FNAC is of great significance for clinical intervention of malignant thyroid lesions. Convolutional neural network (CNN) is a model that can recognize local areas of images. It can extract classification probability information from local image and output the probable classification information in a certain form after comprehensive analysis. Compared with conventional feature extraction model, CNN has a stronger automatic learning ability and higher classification performance and provides a higher accuracy in obtaining information of data with defined features [4–6]. The objective of this study is to investigate the application value of a deep CNN model for cytological assessment of thyroid nodules. Findings from this study will help improve the diagnostic accuracy of malignant thyroid nodules.

## 2. Materials and Methods

### 2.1. Clinical Data

117 eligible patients with thyroid nodules who underwent thyroid cytology examination in the Affiliated People's Hospital of Ningbo University between January 2017 and December 2019 were included in this study. Inclusion criteria: (1) patients whose thyroid nodules need pathological examination by color Doppler ultrasound; (2) patients scheduled to undergo fine-needle aspiration cytology (FNAC); (3) provision of written informed consent. Exclusion criteria: (1) patients with hypertension or diabetes with poor control; (2) patients with autoimmune diseases; (3) patients with malignant tumors in other regions; (4) patients with coagulation dysfunction; (5) patients with acute or chronic infection in recent days; (6) patients who had received a thyroid surgery. This study was reviewed and approved by the Institutional Ethics Committee of The Affiliated People's Hospital of Ningbo University.

### 2.2. Diagnostic Criteria and Outcomes

FNAC results were classified into six grades according to the Bethesda System for Reporting Cervical Cytology [7] proposed by the National Cancer Institute Workshop: I, unsatisfactory specimens or unable to diagnose; II, benign lesion; III, follicular lesion of undetermined significance or atypical cells of undetermined significance (AUS); IV, suspicious follicular tumor or follicular tumor; V, suspicious malignant tumor; VI: malignant tumors. Among them, grades I–IV results indicate nonmalignant lesions, and grades V and VI were malignant lesions. Pathological results showed that FNAC results were malignant in 75 patients and nonmalignant in 42 patients.

### 2.3. Methods

#### 2.3.1. Ultrasound-Guided Puncture and Pathological Smear Preparation

All patients underwent US-FNAC guided by color ultrasound L9-4 high-frequency probe (Sonix SP). They were asked to lie in the supine position with their necks padded up to fully expose the front of the neck. After routine disinfection and local anesthesia with 2% lidocaine, under the guidance of ultrasound, thyroid nodules were sucked using a 22 G × 5 cm needle attached to a 10 ml syringe. For patients with multiple nodules, the nodules with the most malignant signs as indicated by the ultrasound were selected for puncture. The extracts were placed on the slides, pushed or pressed, fixed with 95% alcohol, and stained with hematoxylin/eosin.

#### 2.3.2. Image Preprocessing

100 images of malignant samples and 100 images of nonmalignant samples were captured both at 100×magnification, with reference resolution of 1566 × 1073 dpi (Image Data Generator class in Keras). The training sample images were translated vertically and horizontally. Thus, 900 images were separately created in the vertical and horizontal directions. The sample images were randomly divided into training samples (*n* = 1260) and test samples (*n* = 540) as per the training sample number to test sample number ratio of 7 : 3. Eighty pathological images were collected from patients who received treatment between January 2020 and May 2020 and used as verification set.

#### 2.3.3. Construction of the CNN VGG-16 Model

VGG network was used to investigate the relationship between the depth of CNN and its performance. A 16/9-layer CNN architecture was constructed by repeated stacking of convolution and pooling layers with a kernel size of 3 × 3 and a filter size of 2 × 2. Migration learning was performed based on CNN VGG-16 network, in which 16 represents the number of convolutional layers after excluding pooling layers. Thus, CNN VGG-16 architecture consisted of 13 convolutional layers and 3 fully connected layers (Figure 1). In the first round, two convolutions with 64 kernels were performed, followed by one pooling operation. In the second round, two convolutions with 128 kernels were performed, followed by one pooling operation, then there were two convolutions with 512 kernels, followed by one pooling operation, and finally, there were three full connections. The pretreated images were input into the CNN VGG-16 network, and verification set was input to verify the value of CNN in the screening of malignant thyroid nodules.

#### 2.3.4. Training History and Visualization of Feature Extracts

The dataset was used for training and verification (the ratio was 7 : 3). The test results were obtained after 100 rounds of iteration in terms of accuracy and damage functions. The Gradient-weighted Class Activation Mapping (Grad-CAM) method was used to construct heatmap to locate the areas where the input image contributes greatly to the output by the classification model. The image reading and discrimination ability was compared between the trained CNN dichotomous model and 10 pathologists with more than 5 years of experience in thyroid cell reading and discrimination. The control images were the clinical images collected from 50 patients with malignant or nonmalignant thyroid lesions confirmed by pathological gold standard. One image from one case was selected, thus 100 images were selected.

### 2.4. Statistical Analysis

All experimental data were statistically analyzed using Python 3.6.5 (win64) software. CNN models were established with the Keras library. VGG-16 was used as baseline convolution. Features were extracted from pretrained baseline convolution to achieve optimization.

## 3. Results

### 3.1. Comparison of Patient Data

There were no significant differences in age, sex, body mass index, the diameter of punctured thyroid nodules tumor between malignant and nonmalignant lesion groups (all *P* > 0.05; Table 1).

### 3.2. CNN Model Construction Results

With the increase in the number of iterations, the training and verification loss of CNN model gradually decreased and tended to be stable, and the training and verification accuracy of CNN model gradually increased and tended to be stable. The average loss rate of training samples determined by the CNN model was (22.35 ± 0.62) %, and the average loss rate of test samples determined by the CNN model was (26.41 ± 3.37) %. The average accuracy rate of training samples determined by the CNN model was (91.04 ± 2.11) %, and the average accuracy rate of test samples determined by the CNN model was (91.26 ± 1.02) %. For details, please see Figures 2 and 3.

Typical pathological images of malignant and nonmalignant lesions and the feature images of characteristic kernel generation in VGG-16 model are shown in Figures 4–6.

## 4. Discussion

With the development of digital technology, image-based diagnosis technology has been widely used in clinical diagnosis. But the image capture and retention still depend on the doctor's personal knowledge and experience [8]. Cytological assessment of thyroid gland remains an important method to identify malignant thyroid nodules. This method is greatly limited due to the influence of doctor's personal experience and knowledge. Therefore, its values in the identification of malignant thyroid nodules are likely different and limited to a certain degree [9–11].

In recent years, with the development of digital technology and deep learning network, medicine and digital technology are closely linked. A network model has been proposed for the diagnosis and prediction of various diseases and some achievements have been made [12, 13]. The CAD system can be used as an additional expert in the double screening process to improve human diagnostic performance based on computer programs. This system helps doctors to diagnose diseases by applying and processing one or more medical images collected. It has been widely used for the diagnosis of brain, breast, lung and thyroid diseases [14, 15]. CNN is a network system with extraordinary visual recognition ability. The accuracy of CNN model constructed based on residual neural network (ResNet) architecture in large-scale visual recognition challenge task is 96.4%, which is higher than 94.9% provided by human [16]. ResNet can solve the problem that gradiently disappears when there are too many network layers by introducing residuals into the network. It can construct ResNet neural network at different depths by combining and stacking the residuals.

In this study, we analyzed the data of patients who received cytological assessment of thyroid gland in The Affiliated People's Hospital of Ningbo University. Our results showed that among the 117 patients included in this study, 75 had malignant thyroid nodules. We established CNN-CAD model of thyroid nodules and performed deep training and data verification. We found that the average accuracy and average loss rate of training samples in the CNN model in the identification of malignant thyroid nodules were (91.04 ± 2.11) % and (22.35 ± 0.62) %, respectively, and they were (91.26 ± 1.02) % and (26.41 ± 3.37) % respectively for the test samples. With the increase in the number of iterations, the training and verification loss of CNN model gradually decreased and tended to be stable, and the training and verification accuracy gradually increased and tended to be stable.

Our results showed that the accuracy of CNN model in the identification of malignant thyroid nodules was closely related to the size of Epoch. A smaller number of Epoch leads to low learning ability of the CNN model, producing greater diagnostic or prediction deviation, and finally resulting in lower accuracy of CNN model in the identification of malignant thyroid nodules. If the number of Epoch is too high, CNN model can converge after a certain number of iterations. This can increase the recognition rate but also leads to overfitting due to the increase of model training time. When the number of Epoch is 100, the CNN model can fully learn the training dataset without over convergence. When the number of convolutional kernels is too small, the ability of CNN model to extract features is correspondingly low. With the increase of the number of filters, its accuracy increases in the identification of malignant thyroid nodules. With the continuous increase of filter numbers, the number of parameters to be trained and the time of training and recognition in the CNN network will also increase. When the feature extraction has reached the maximum, its accuracy tends to be stable and does not change.

Taken together, the models for cytological identification of malignant thyroid nodules, constructed based on CNN, are of auxiliary value in the diagnosis of malignant thyroid nodules. Perrin [17] and Li [18] used deep CNN to segment liver tumors and achieved a higher accuracy in identifying malignant liver tumors. All these findings confirm that deep CNN has good classification performance and automatic learning ability and can accurately describe the potential information of dataset. However, this is a single-center study with a relatively small sample size. This study did not effectively analyze the ethnic, regional, and other factors. A single-center study may have some restrictions on the consideration of treatment method and other factors. In addition, retrospective analysis can make research information biased. Therefore, the results may be slightly different from the actual phenomenon. Multicenter studies involving larger sample sizes are needed to adequately address the limitations this study posed.

## Figures and Tables

**Figure 1:** Architecture diagram of the VGG-16 model.

**Figure 2:** Training and testing loss for the convolutional neural network (CNN) model.

**Figure 3:** Training and test accuracy for the convolutional neural network (CNN) VGG-16 model.

**Figure 4:** Pathological image of typical nonmalignant lesion.

**Figure 5:** Pathological image of typical malignant lesion.

**Figure 6:** Images of characteristic kernel generation in the first five layers in the VGG-16 model.

**Table 1:** Comparison of patient data.

General data	Malignant lesion (*n* = 75)	Nonmalignant lesion (*n* = 42)	*χ* ^2^ */t*	*P* value
Age ($\bar{\chi }$ ± *s*; year)	43.56 ± 11.89	42.74 ± 12.03	0.356	0.722
Sex (*n*)				
Man	15	5	1.245	0.265
Women	60	37		
Body mass index ($\bar{\chi }$ ± *s*; Kg/m^2^)	23.15 ± 3.02	22.98 ± 3.11	0.289	0.773
Diameter of punctured thyroid nodules ($\bar{\chi }$ ± *s*; cm)	0.452 ± 0.05	0.47 ± 0.08	1.664	0.099

## Data Availability

The simulation experiment data used to support the findings of this study are available from the corresponding author upon request.

## Additional Points

As shown in Figure 6, with the increase in the number of layers of the CNN-VGG-16 model, the cytological features of thyroid nodules become more obvious. When the number of layers was too high, the image was distorted and mosaic changes appeared.
